The article "A Novel Psychotherapy Effect Detector of Public Art Based on ResNet and EEG Imaging" was published in 2022. Journal: Comput Math Methods Med.

# A Novel Psychotherapy Effect Detector of Public Art Based on ResNet and EEG Imaging

**DOI:** 10.1155/2022/4909294

**Published:** 2022-04-07

**Authors:** Tingyi Tian, Le Wang, Man Luo, Wei Zhu

**Affiliations:** ^1^School of Art and Design, Shanghai University of Engineering Science, Shanghai 201620, China; ^2^Department of Design, National Taiwan Normal University, Taipei, Taiwan; ^3^Product Design and Development Laboratory, Taiwan

## Abstract

**Methods:**

The EEG emotion dataset seed is used for feature extraction with DE, and the emotion is recognized by ResNet. Adam optimizer is used to classify the extracted DE through ResNet50 model. Each batch is set as 5 groups of data and is trained for 50 rounds, then the model is optimized, and the accuracy rate is 76.47%, which output the probability of good emotion through the model. We put the model optimized by ResNet into the intelligent module and visualize it with numerical value.

**Results:**

The detector designed by EEG data and ResNet50 optimization model has high accuracy. The results show that the error between the detector data and the questionnaire interview data is small, the average error is 2.77, and the accuracy is 97%. The closer the subject's emotion before the test is to neutral emotion, the closer the questionnaire result is to the test result of the tester, and the smaller the error is. The difference between the tester data and the survey questionnaire data is 0.2, which is in good agreement and has small error. It can be seen that the detector has high accuracy.

**Conclusion:**

Our proposed public art psychotherapy effect detector has good accuracy in detecting users' emotions. It can detect the group psychotherapy effect of public art and can classify and screen a large number of public arts in the city by quantitative methods. It provides support for further summarizing the practical utility of public art and provides a new way for the optimal design and follow-up evaluation of public art design.

## 1. Introduction

The development of public art today has developed greatly in both scale and quality. In recent years, public art has become an important part of people's living space because of its characteristics of multilevel, multistage, multiconnotation, multiform, and participation. More than 300 cities in North America will legislate for public art. With the complexity and diversification of social needs, public art research began to focus on exploring its effectiveness in the regulation and relief of spirit and emotion. Human participation in creative cultural activities is conducive to mental health and emotional regulation, as well as the transmission of health information and the enhancement of social tolerance [1]. Participatory art also has potential benefits for mental health [2]. Participation is not only a way to express and release but also a way for people to adjust their inner emotions and change space scenes. In the production of public art, it forms resonance based on human emotion [3]. This empathy and resonance are a means for public art to have an impact on people's spirit and psychology. Moreover, public art has the function of social psychological intervention. It stimulates the public's psychological reflection and acceptance through some art form. Many theoretical studies have proved that public art has a certain effect on emotional regulation and psychotherapy.

The article "A Novel Psychotherapy Effect Detector of Public Art Based on ResNet and EEG Imaging" was published in 2022. Journal: Comput Math Methods Med.

The evaluation of public art psychotherapy effect has been a qualitative study in previous studies. Most are evaluated by artists, designers, or government departments and organizations that invest in public art. The feedback by public participation is basically in the form of interview, which is highly subjective. More subjective evaluation is not conducive to the establishment of evaluation system and the optimization of public art design principles. With the rapid development of artificial intelligence, emotion recognition computing technology can recognize the changes of emotion from the technical level and classify. Emotion is people's attitude experience and corresponding behavior response to objective things. It is also a psychological phenomenon mediated by individual needs, wishes, and other tendencies [4].

Therefore, identifying people's emotions when participating in public art can evaluate public art more objectively. In emotion recognition, micro expression information, language voice, posture expression, and physiological signals are important data sources [5]. Among these data sources, EEG signal is the most typical physiological signal, which is difficult to disguise and rich in information. EEG signal is the overall response of electrical activities of nerve cells in the cerebral cortex or scalp surface, which contains a lot of physiological and pathological information [6]. The fluctuation of emotion will have an impact on the physiological signals of the body and will inevitably have a corresponding impact on the brain waves [7]. Therefore, by collecting and analyzing EEG signals, we can intuitively and accurately judge the physiological and psychological state of the human body. Lin et al. [8] used convolutional neural network to collect a variety of human physiological parameters through wearable devices and tried to send different control commands to the manipulator according to the changes of emotion. Naima and Canny [9] detected human EMG, ECG, blood oxygen saturation, respiratory rate, and exercise status through wearable devices and used artificial intelligence technology to realize real-time monitoring of personal physical and mental health. Pan et al. [10] trained the model based on EEG signals and convolutional neural network to classify emotions. The key problem of EEG signal analysis is feature extraction. In emotion recognition, EEG signal features are mainly extracted from time-domain features [11], frequency-domain features [12], time-frequency-domain features [13], nonlinear dynamic analysis [14], spatial domain features [15], and so on. At the same time, in previous studies, sensor-based consciousness and emotion awareness basically realized an efficient and natural human-computer interaction [16]. However, there is little research on the application of this method in the field of public art.

The article "A Novel Psychotherapy Effect Detector of Public Art Based on ResNet and EEG Imaging" was published in 2022. Journal: Comput Math Methods Med.

This paper attempts to solve the problem that the public's evaluation on public art stays at the stage of large subjective factors, which is based on the research basis of emotion recognition and classification by the combination of artificial intelligence and sensors, so as to make it have an objective and quantitative evaluation method. Therefore, this paper proposes to collect EEG data, analyze the data through convolution neural network and ResNet model, and visualize human-computer interaction, so as to complete the detection of public art psychotherapy effect and achieve the objectivity of public art social evaluation at the same time. The public art psychotherapy effect detector designed in this paper not only provides a scheme for the measurement of the practical utility of public art but also provides a method for the evaluation of a large number of existing public art in the city, so as to promote the design of public art to have more practical effects.

## 2. Methodology

### 2.1. Residual Neural Network

Residual neural network [17] has achieved excellent results in many competitions in the field of visual recognition. We know that the greater the complexity of the model is, the higher the accuracy will be, but this does not mean that the more complex the model is, the higher the efficiency of improving the accuracy will be. “Moore's law” [18] also appears in deep learning, that is, with the increase of the number of layers of the model, it will cost more to improve the accuracy a little later. Because with the increase of the number of model layers, it is bound to bring huge consumption of computing resources, and there will be the problem of “gradient disappearance.”

ResNet solves the problem of “gradient disappearance” [19] which is also an important reason why this paper uses ResNet for experiments. ResNet is developed on the basis of VGG19. It adds residual unit through short circuit mechanism, directly uses convolution with step size of 2 for down sampling, and replaces the full connection layer with Global Average Pooling (GAP) layer. In the ResNet model, two residual elements are mainly used, as shown in Figure 1. The build block on the left corresponds to the shallow network, while the bottleneck block on the right corresponds to the deep network. There are two paths for the input information. The first is identity mapping. Identity mapping ensures that the learned information is completely saved. If improvement is needed, it is carried out in the direct mapping, that is, *f*(*x*) In. The better *f*(*x*) changes the information between blocks, the better the performance of the model.

The article "A Novel Psychotherapy Effect Detector of Public Art Based on ResNet and EEG Imaging" was published in 2022. Journal: Comput Math Methods Med.

The purpose of residual structure is to make the neural network retain the ability of basic identity mapping. This ability can ensure that the network training results will not degrade with the stacking of networks. Assuming that the input parameter of the neural network is *x*, the target output is *h* (*x*), and the internal structure of *H* (*x*) may not be clearly expressed. ResNet allows the residual *f* (*x*) = *H* (*x*) − *x* directly learned by the submodule to make the target output *F* (*x*) + *X*, which avoids the performance degradation and accuracy degradation caused by too many convolution layers. The structure on the right belongs to the shortcut connection. Through the shortcut operation before activating the function, add the output before this layer and the output after passing through the network of this layer, and send the added value to the activation function to obtain the total output of this layer. ResNet has a shortcut connection; assuming that the input is *x*, the output *y* is

(1) $$\begin{array}{c} y=F\left(x,\left\{W_{i}\right\}\right)+x. \end{array}$$

The relationship between the normal data input and the output obtained by the neural network is as follows. Since there is an activation function ReLU in the middle, considering the double-layer weight, there are

(2) $$\begin{array}{c} F=W_{z}\sigma \left(W_{1}x\right). \end{array}$$

Generally, the activation function ReLU is used to increase the nonlinearity and associate the weights *W*1 and *W*2 of the function and structure layers. Changing the number of channels can change the dimensions of the input data and output data of the signal. Here, when shorting, make a linear transformation WS for *X*, as follows:

(3) $$\begin{array}{c} F=W_{z}\sigma \left(W_{1}x\right). \end{array}$$

In this paper, ResNet50 network model is selected for image feature extraction, precisely because ResNet network has long been widely used in image feature extraction in various fields, and the residual module in ResNet50 residual neural network can effectively solve the degradation problem with the deepening of the network, as well as the problem of insufficient learning ability of the model with shallow network layers and poor effect of feature extraction.  Figure 2 is a structure diagram of ResNet50 network. The whole network structure is divided into 50 layers and consists of four large modules: the first large module has three small modules, the second large module has four small modules, the third large module has six small modules, and the fourth large module has three small modules, in which each small module is composed of three convolution cores. The convolution layer of the first layer and the full connection layer of the last layer of the network are added to constitute a 50-layer network structure.

The article "A Novel Psychotherapy Effect Detector of Public Art Based on ResNet and EEG Imaging" was published in 2022. Journal: Comput Math Methods Med.

### 2.2. EEG Sensor Data Acquisition

Emotion recognition of EEG signals mainly includes five basic steps [20], as shown in Figure 3.

EEG signal is an extremely weak physiological signal (with amplitude at microvolt level). In the acquisition process, it will not only be disturbed by EEG data acquisition equipment and external environment but also be affected by some physiological factors of the human body, such as eye electricity and electromyography [21]. At the same time, the current physiological and psychological state of the tester will also affect the acquisition of EEG signals. A large number of artifact signals will increase the difficulty of EEG signal analysis, and it is difficult to intuitively analyze the internal relationship with emotion. In order to facilitate the follow-up research, the collected signals are preprocessed. Through this preliminary processing, the signals with certain laws can be obtained [22].

### 2.3. Database

SEED [23] public database was used in this experiment [24]. This dataset has the largest number of EEG acquisition channels, with 62 channels of EEG collected from 15 subjects. Participants were asked to watch a video of positive/negative/neutral emotions for about four minutes each, and the corresponding electrical signals were recorded. The dataset has a longer duration used for emotionally stimulating videos, which is more conducive to the emotional expression of subjects, and its classification accuracy is higher than other public databases.

The database data were obtained by selecting 15 film clips (positive, neutral, and negative emotions) from the library as stimuli used in the experiment. Stimulants (film clips) were selected according to the following criteria: (a) the length of the entire experiment should not be too long to avoid subject fatigue; (b) the video can be understood without explanation; (c) the video should elicit a single target emotion. Each film clip lasts about four minutes, and each film clip is carefully edited to create coherent emotion and maximize emotional meaning [25]. There were 15 experiments in each experiment. There is a 5-second prompt before each clip, a 45-second self-assessment, and a 15-second break after each clip in a session. The order of presentation is arranged in such a way that two movie clips targeting the same emotion are not played consecutively. To get feedback, participants were told to report their emotional response to each film clip by completing a questionnaire immediately after watching each clip [26]. The detailed process is shown in Figure 4.

The article "A Novel Psychotherapy Effect Detector of Public Art Based on ResNet and EEG Imaging" was published in 2022. Journal: Comput Math Methods Med.

In the SEED database's “Preprocessed_EEG” folder, there are files that contain downsampled, preprocessed, and segmented versions (.mat) of EEG data in MATLAB. The data is downsampled to 200 Hz. A bandpass frequency filter of 0-75 Hz is applied. In this design, EEG segments corresponding to the duration of each film were extracted. There are 45 .mat files (MATLAB files), in which one file matches each experiment. Each subject underwent 3 experiments, with an interval of about 1 week. Each topic file contains 16 arrays. The 15 arrays contain segmented preprocessed EEG data (EEG_1 to EEG_15, channel × data) for 15 trials in one experiment. The array name tag contains the tag for the corresponding emotion tag (-1 for negative, 0 for neutral, and +1 for positive). The detailed order of channels is contained in the dataset, as shown in Figure 5.

SEED data is an EEG dataset used to analyze human emotion. The dataset collected and recorded the EEG signal data of 15 human subjects (7 males and 8 females) when they watched videos with obvious emotional stimulation effect for about 4 minutes, so as to analyze the relationship between their emotional changes and EEG signal. In order to ensure the reliability of the test results, 15 subjects were tested in three different periods of time, watching 15 videos, respectively, in each test, and recording the changes of EEG signals. Related data were extracted by MATLAB software, and PS, DDE, DASM, RASM, ASM, and DCUA data were obtained. Previous studies have proved that DE (differential entropy) data has the highest accuracy in emotion recognition [24], so this paper adopts DE data in SEED data for modeling. DE can be expressed by the formula

(4) $$\begin{array}{c} h\left(X\right)=-\int_{-\infty }^{\infty }\;\frac{1}{\sqrt{2\pi \sigma^{2}}}e^{-{\left(x-\mu \right)}^{2}/2\sigma^{2}}\log\left(\frac{1}{\sqrt{2\pi \sigma^{2}}}e^{-{\left(x-\mu \right)}^{2}/2\sigma^{2}}\right)dx=\frac{1}{2}\log\left(2\pi e\sigma^{2}\right). \end{array}$$

The time series *X* obeys the Gaussian distribution *n*(*μ*, *σ*^2^). In order to remove the components irrelevant to emotion, the linear dynamic system (LDS) [25] method with a window length of 20 s is used to smooth the feature sequence. The data dimension is 62 × *N* × 5, where 62 represents 62 regions of the brain, *N* is the length of EEG signal, and 5 represents the corresponding five bands (delta: 1-3 Hz, theta: 4-7 Hz, alpha: 8-13 Hz, beta: 14-30 Hz, and gamma: 31-50 Hz). In this paper, *N* = 180 is uniformly used, that is, the dimension of DE_LDS dataset is 62 × 180 × 5. Finally, the data is unified to reshape a two-dimensional data 224 × 224. A total of 675 groups of sample data of DE_LDS were obtained. In order to train the model, 675 groups of data were randomly allocated according to the ratio of 9 : 1 between training set and test set, which get 607 training sets and 68 test sets. The model is trained on the training set and the accuracy of the model is tested on the test set.

The article "A Novel Psychotherapy Effect Detector of Public Art Based on ResNet and EEG Imaging" was published in 2022. Journal: Comput Math Methods Med.

#### 2.3.1. Standardization

Before entering the model, the data needs to be standardized. In this paper, the minimax standardization method is used to unify the data at the same dimensional level [19]. The formula is as follows:

Pair and sequence *x*_1_, *x*_2_, *x*_3_, ⋯, *x*_*n*_:

(5) $$\begin{array}{c} \;y_{i}=\frac{x_{1}-\min\left\{x_{1},x_{2},x_{3},\cdots ,x_{n}\right\}}{\max\left\{x_{1},x_{2},x_{3},\cdots ,x_{n}\right\}-\min\left\{x_{1},x_{2},x_{3},\cdots ,x_{n}\right\}}. \end{array}$$

New sequence *y*_1_, *y*_2_, *y*_3_, ⋯, ∈[0, 1].

#### 2.3.2. Loss Function

In the classification task, the loss function mainly used in this paper is the categorical_crossentropy loss, which is defined as

(6) $$\begin{array}{c} C=-\frac{1}{n}\underset{x}{\sum }\left[y\ln a+\left(1-y\right)\ln\left(1-a\right)\right], \end{array}$$

where “*y*” is the desired output and “*a*” is the actual output of the neuron.

#### 2.3.3. The Activation Function

Activation function is responsible for mapping the input of neurons to the output, which plays a very important role in the fitting of deep learning model. The activation functions mainly used in this paper include ReLU function and Softmax function.

The ReLU function is used in the hidden layer of the model to speed up the learning of the model. Its mathematical formula is as follows:

(7) $$\begin{array}{c} \text{ReLU}\left(x\right)=\left\{\begin{array}{cc} x & x>0,\\ 0 & x<=0. \end{array}\right. \end{array}$$

Softmax function is used for the final output of the model. It maps the output of multiple neurons to the (0, 1) interval to carry out multiclassification. Its mathematical formula is as follows:

(8) $$\begin{array}{c} \text{Softmax}\left(x_{i}\right)=\frac{\exp\left(x_{i}\right)}{\sum_{j=1}^{n}\exp\left(x_{j}\right)}, \end{array}$$

where “*x*_*i*_” is the output value of the node and “*n*” is the number of output nodes, that is, the number of categories classified. Through the Softmax function, the output values of multiple classifications can be converted into probability distributions ranging from [0, 1] to 1.

The article "A Novel Psychotherapy Effect Detector of Public Art Based on ResNet and EEG Imaging" was published in 2022. Journal: Comput Math Methods Med.

### 2.4. Human-Computer Interaction (HCI) Detection Design

In this design, EEG wearable devices are used to collect electrical signals from the brain. The sensor module is just like neurons on the human body, sensing the stimulation of external substances all the time. The specific measurement process of this design is as follows: it sets the whole measurement time for 60 s and controls the red light in the sensor to emit light at 200 Hz in the first 30 s, which starts collecting EEG signals at a sampling rate of 200 Hz, that is, collects a signal point every 5 ms and stores the brainwave signals. The working process of the last 30 s is that the EEG signal is transmitted to the human-machine interface module through Bluetooth, and the human-machine interface analyzes and visualizes the data collected by the sensor. The detection workflow is shown in Figure 6.

#### 2.4.1. The Sensing Module

Sensor module is the basis of human-computer interaction and an important part. It includes power module, EEG sensor device, intelligent module, and Bluetooth module. The system structure is shown in Figure 7.

#### 2.4.2. Human-Machine Interface

In the HCI interface, based on the intelligent module, the data samples were extracted from the difference entropy (DE) feature and analyzed in the emotion classification model module by preprocessing the collected data. The design established the emotion classification model module through the ResNet50 model and SEED public database to achieve the emotion classification and visual display to detect the user's emotional state. HCI interface is shown in Figure 8.

## 3. Results

### 3.1. ResNet50 Network Training

In this paper, Adam optimizer is used, and the learning rate is set as the default parameter. By entering the data into the model in batches, each batch is set as 5 groups of data, and a total of 50 rounds are trained. After each round, the accuracy test (accuracy) of the model is carried out through the test set, in which the accuracy changes with rounds, as shown in Figure 9.

The experimental results show that the model with the highest accuracy rate is the 39th round of training, and its accuracy rate can reach 0.7647. Therefore, the 39th round model is finally determined as the final model in this design. For better visualization, in the model, the higher the probability is set, the higher the pleasure is, which is a good emotion. The lower the probability is set, the lower the degree of pleasure is, which is a bad emotion, and the middle value is neutral emotion.

The article "A Novel Psychotherapy Effect Detector of Public Art Based on ResNet and EEG Imaging" was published in 2022. Journal: Comput Math Methods Med.

### 3.2. Human Testing Experiment

The detector can detect in the normal active state of nonstationary, but it is not suitable for detection in the state of running and vigorous exercise. Five public arts in Shanghai were selected for the test experiment, as shown in Table 1. These public arts chosen for the test are the works in Shanghai's 2019 and 2021 city space art season, which has the most reading volume on the WeChat official account. Before the experiment, 30 questionnaires were conducted on the pleasure degree generated by the five public art projects. The pleasure degree was set to 1-100. The higher the value is, the higher the pleasure degree is. A total of 28 valid questionnaires were collected and averaged. The survey results show that among the five public arts, public art no. 1 has the highest pleasure, with a value of 82. The public art is set in the community and has strong participation; public art no. 5 has the lowest pleasure with a value of 70. This public art is a large sculpture in Yangpu Binjiang Park. The pleasure degree of each public art project is shown in Figure 10.

Another 6 people were tested to wear the detector. The subjects were between 25 and 40 years old. The nature of work was civil servants, public institutions, teachers, financial industry, and computer industry, and everyone wore the detector one time in work or life before the experiment. They wore the detector once when appreciating or participating one of the five public arts selected in the experiment. The value displayed by the tester was 1-100. The higher the value is, the higher the pleasure is. The two rounds of test results are shown in Figure 11.

The experimental results show that the error between the test data and the questionnaire interview data is small, the average error is 2.77, and the accuracy is 97%; it shows that the accuracy of the tester is high. In the experiment, the closer the subjects' emotion before the test is to neutral emotion, the closer the questionnaire results are to the test results of the detector, and the smaller the error is. According to the data of the tester, the average pleasure improvement value of 6 subjects in public art no. 1 is 34.2, and the average pleasure improvement value of public art no. 5 is 22, with a difference of 12.2. The results of the questionnaire show that the average pleasure of no. 1 public art is 82 and that of no. 5 public art is 70 with a difference of 12. It can be seen that the error between the experimental results and the results of the questionnaire is small, and the difference is 0.2.

The article "A Novel Psychotherapy Effect Detector of Public Art Based on ResNet and EEG Imaging" was published in 2022. Journal: Comput Math Methods Med.

## 4. Discussion

In the past, public art was mainly evaluated from the perspective of designers, artists, and government investors. There are fewer evaluations from the public, and the evaluations mainly adopt the form of interview, which was highly subjective. And there is no measurable method to determine whether a large number of public arts in cities have practical utility. The public art psychotherapy effect detector based on ResNet network and EEG sensor designed in this paper can collect more objective people's feelings about public art and classify the good, neutral, and bad emotions generated by public art through emotion recognition, which evaluates the public art psychotherapy effect at the same time. Therefore, it has certain innovation.

The model designed in this paper adopts SEED public data, which is optimized by ResNet50 model, ReLU function and Softmax function activation, and Adam optimizer. Finally, the intensive reading of model recognition reaches 76.47%.

The psychotherapy effect of public art can be tested by comparing the data wearing the detector in normal state with the data when participating in public art. Although individual differences and the emotional state before the test are variable factors, the detector shows high accuracy by comparing the test results of the same public art with the questionnaire results of different subjects, Therefore, the effects of different public art psychotherapy can be tested. In addition, by comparing the test results of different public arts with the questionnaire results of the same subjects, the detector also showed high accuracy. Therefore, the psychological healing effects of different public arts can be evaluated and analyzed, which has certain practicability.

The detector designed in this paper also has some limitations. First, the model training uses a public database, so the data acquisition of the detector needs to use the same acquisition channel as the data of SEED database. Second, this experiment analyzes EEG data, but other physiological data can also carry out emotion analysis, but multisensor will bring greater difficulty to data analysis. In the follow-up upgrading research of detector, we will try to use multisensor.

## 5. Conclusion

The development of efficient machine learning algorithms and the creation of ubiquitous wearable technologies make emotional interaction possible and have a quantifiable and detectable data acquisition method. The public art psychotherapy effect detector based on ResNet network and EEG sensor has good accuracy in detecting users' emotions and can detect the group psychotherapy effect of public art. Therefore, it can classify and screen a large number of public arts in the city by quantitative methods. It provides support for further summarizing the practical utility of public art and provides a new way for the optimal design and follow-up evaluation of public art design.

The article "A Novel Psychotherapy Effect Detector of Public Art Based on ResNet and EEG Imaging" was published in 2022. Journal: Comput Math Methods Med.

## Figures and Tables

**Figure 1:** Two residual elements.

**Figure 2:** ResNet50 network architecture.

**Figure 3:** Main steps of EEG emotion recognition.

**Figure 4:** SEED data acquisition experiment process.

**Figure 5:** International standard 10-20 system 62-channel EEG.

**Figure 6:** Workflow of detector.

**Figure 7:** Sensor module system structure.

**Figure 8:** Human-machine interaction interface design description: (a) main interface; (b) charging interface; (c) user information interface; (d) system setting interface.

**Figure 9:** Variation of test accuracy with training epoch.

**Figure 10:** Survey results.

**Figure 11:** Results of two rounds of data of 6 subjects.

**Table 1:** List of selected public art projects.

Number	Name of public art
1	Siping Road “poetry one-way street”
2	Xinhua community public art
3	Public art of Caoyang Baixi Park
4	A move in Linfen community
5	Yangpu Binjiang public art “things outside the sky”

## Data Availability

Data are available on request from the authors due to privacy/ethical restrictions.
